The article "A New Generation of ResNet Model Based on Artificial Intelligence and Few Data Driven and Its Construction in Image Recognition Model" was retracted in 2023. Reasons: unreliable results or conclusions; concerns about the data; concerns about the results or conclusions; concerns about the peer review.

# A New Generation of ResNet Model Based on Artificial Intelligence and Few Data Driven and Its Construction in Image Recognition Model

**DOI:** 10.1155/2022/5976155

**Published:** 2022-03-19

**Authors:** Hao Wang, Ke Li, Chi Xu

**Affiliations:** ^1^Shandong Anhui Information Technology Co., Ltd., Jinan 250100, Shandong, China; ^2^Shandong Anyong Precision Machinery Co., Ltd., Taian 271000, Shandong, China; ^3^Shandong Kangyuan Technology Innovation Development Co., Ltd., Jinan 250100, Shandong, China

## Abstract

The paper proposes an A-ResNet model to improve ResNet. The residual attention module with shortcut connection is introduced to enhance the focus on the target object; the dropout layer is introduced to prevent the overfitting phenomenon and improve the recognition accuracy; the network architecture is adjusted to accelerate the training convergence speed and improve the recognition accuracy. The experimental results show that the A-ResNet model achieves a top-1 accuracy improvement of about 2% compared with the traditional ResNet network. Image recognition is one of the core technologies of computer vision, but its application in the field of tea is relatively small, and tea recognition still relies on sensory review methods. A total of 1,713 images of eight common green teas were collected, and the modeling effects of different network depths and different optimization algorithms were explored from the perspectives of predictive ability, convergence speed, model size, and recognition equilibrium of recognition models.

## 1. Introduction

Green tea is good for people's physical and mental health and is a popular beverage among consumers. At the same time, green tea is also the most diverse and the most produced tea in China, and appearance is an important basis for its classification and differentiation of grades, as well as an important part of team sensory evaluation. However, the traditional tea sensory review method uses review terminology that has not been perfected [1]. The uncertainty of the objective environment, the low prevalence of standard quantities, the interference of subjective factors by tea evaluators, the poor repeatability, and other limitations do not match the increasing consumer demand for accurate information and safe and high quality tea products in the current new era [2]. Therefore, the development of open, standardized, and intelligent [3] green tea classifications and identification methods is an inevitable trend. New classification and assessment methods for green tea have been emerging, such as physicochemical review methods [4, 5], fingerprinting assessment methods [6, 7], intelligent sensory review methods [8, 9], and infrared spectral imaging technology detection methods [10, 11], but these methods have their limitations to a certain extent, such as relevant instruments and cumbersome and complicated operations, and most of them are based on the overall tea leaves. It is necessary to propose an objective, simple, fast, and low-cost method for green tea classification, since most of them are based on the whole tea leaves for review, which requires specific and time-consuming requirements.

The article "A New Generation of ResNet Model Based on Artificial Intelligence and Few Data Driven and Its Construction in Image Recognition Model" was retracted in 2023. Reasons: unreliable results or conclusions; concerns about the data; concerns about the results or conclusions; concerns about the peer review.

Convolutional neural networks, as an important member of image classification algorithms, have the advantages of high recognition accuracy, fast detection speed, and great development potential [12], have achieved considerable success in image classification [13], object detection [14], pose estimation [15], image segmentation [16], and face recognition [17, 18], have great scaling advantages [19], and have been widely used in agriculture [20], healthcare [21], education [22], energy [23], industrial inspection [24], and other fields [25]. Currently, convolutional neural networks have been used for tea tree pest and disease identification [26], tea grade sieving [7], and the sorting of tea tree fresh leaves [8], but for the recognition and classification of different species of green tea based on ResNet, a typical convolutional neural network is proposed by researchers in recent years to perform computer vision tasks, which minimizes the gradient disappearance problem caused by increasing the depth of the network due to the introduction of the residual module and reduces the redundancy of information in the data while maintaining a high accuracy rate, which is simple and practical.

Based on ResNet convolutional neural network, this study constructs a deep learning model capable of distinguishing 8 kinds of green tea by selecting the appropriate optimization algorithm and model depth, aiming to develop an efficient, accurate, and objective identification model and apply it to mobile, realizing the recognition of green tea pictures in different backgrounds and environments, which can be shared and used by multiple people and devices, saving resources and realizing deep learning in tea recognition. The identification of green tea is a new way of thinking.

## 2. Materials and Methods

### 2.1. Data Acquisition and Test Platform Construction

The dataset of this study consists of 8 kinds of green teas, such as Lishui fragrant tea, Xinyang Maojian, Lu'an Guapian, Taiping Monkey Kui, Anji White Tea, Biluochun, Bamboo Leaf Green, and Longjing. The number of images of each kind is shown in Table 1, with a total of 1,713 images. Part of the dataset of this study is shown in Figure 1. The eight kinds of green tea with different appearance and quality characteristics present different states in different scenes with different backgrounds, which better reproduce the actual scenes of tea in life. These images are manually searched from different Internet platforms, such as the shopping platform Jingdong (https://www.jd.com), Tao Bao (https://www.taobao.com), the social platform Weibo (https://weibo.com), and Baidu Post (https://tieba.baidu.com), with different brightness, background, and angle. The higher the resolution of the image is, the more features it contains, and the better it is for model learning. Therefore, the image datasets selected in this study are basically above 100 KB in size, and extended formats are basically JPG and PNG.

The article "A New Generation of ResNet Model Based on Artificial Intelligence and Few Data Driven and Its Construction in Image Recognition Model" was retracted in 2023. Reasons: unreliable results or conclusions; concerns about the data; concerns about the results or conclusions; concerns about the peer review.

The experimental platform for this study was built as shown in Table 2, and the modeling scripts used are available on github (https://github.com/seldas/DL_Beetles).

### 2.2. Image Preprocessing

The original images obtained in this study vary in size, and conducting some preprocessing of the images can enhance the recognition of the target objects by the model and also avoid overfitting of the network. In this study, the tea images in the training set were first randomly cut into RGB images in the image format of 224 × 224 × 3 and then flipped. The images in the test set are first scaled and then cropped to 224 × 224 × 3 RGB images with the center as the reference. In this study, the preprocessing of the images in the test is a data enhancement operation, which can effectively improve the fitting ability and generalization ability of the model [9].

### 2.3. Data Processing and Evaluation Indicators

The images were randomly selected and sampled according to the training set : validation set = 3 : 1. The training data were used for parameter learning, and the validation data were used for model performance evaluation. The same preprocessing was strictly followed, and to ensure the accuracy of the validation results, each set of experiments was repeated at least three times, cross-validation was adopted to avoid the arbitrariness in dividing the training and test sets, and the data were analyzed by one-way ANOVA (*p* < 0.05) using SPSS 21.0 software for significant differences, and finally the data were divided into batches of the same size The data were divided into equal-sized batches to facilitate subsequent model training.

In order to evaluate the performance of ResNet model for green tea species classification, accuracy, error rate, precision rate, recall rate, F-value, and the confusion matrix were adopted as the evaluation indexes in this experiment. Taking the eight types of green tea in this study as an example, the accuracy rate is the average of the overall performance of the model in recognizing the eight types of green tea, and the error rate corresponds to the accuracy rate, which can be suitable for the comparison of recognition balance because of its small base. Accuracy, recall, and *F*-value are performance evaluations for each of these categories. Taking Anji white tea as an example, the accuracy rate is the proportion of all samples predicted to be Anji white tea which are predicted correctly; the recall rate is judged on the basis of samples whose true label is Anji white tea, and it is the proportion of those predicted correctly to all samples whose true label is Anji white tea; and the F-value is a composite index, which is the summed average of the accuracy rate and recall rate. The confusion matrix can summarize and compare the classification prediction results and the actual target, and from the presentation in the form of *N* × *N* matrix, the sum of each row is the number of real samples of the category, and the sum of each column is the number of samples predicted as the category, which can directly evaluate the effectiveness of the classification method.

The article "A New Generation of ResNet Model Based on Artificial Intelligence and Few Data Driven and Its Construction in Image Recognition Model" was retracted in 2023. Reasons: unreliable results or conclusions; concerns about the data; concerns about the results or conclusions; concerns about the peer review.

## 3. Related Theories

### 3.1. Traditional ResNet Network Structure

Since Alexnet [11], the CNN structure has been deepening, and VGG and GoogLeNet [12] have 19 and 22 convolutional layers, respectively. With the increase of network depth, the existence of gradient disappearance problem makes the network training more difficult and the convergence result is not good, and then the ResNet network [13] is introduced, as shown in Figure 2.

The output of the residual module in ResNet is obtained by summing the backbone network with the jump connection, and the shortcut connection adopts a constant mapping. ResNet network can better weaken the gradient disappearance phenomenon, retain more original information in the input image, reduce the loss, and also improve the convergence speed in deeper networks compared with the traditional VGG network, essentially reducing the training. The redundancy of data information in the training process is essentially reduced, but the shortcut direct connection makes it less focused on the local target information in multiple categories, which reduces the classification accuracy.

### 3.2. Dropout Layer

The dropout layer is a layer that is used to temporarily discard neurons with a certain probability during the training process of the network. When the data samples are small, it can prevent the model from overfitting and effectively improve the classification accuracy. Reference [14] introduced the dropout layer into the convolutional neural network, which not only solved the overfitting phenomenon but also obtained good classification accuracy.

The article "A New Generation of ResNet Model Based on Artificial Intelligence and Few Data Driven and Its Construction in Image Recognition Model" was retracted in 2023. Reasons: unreliable results or conclusions; concerns about the data; concerns about the results or conclusions; concerns about the peer review.

### 3.3. Residual Attention (Attention) Network

Attention networks can highlight local target information and allow the network to focus more on finding useful information related to the output in the input image, thus improving the classification accuracy of image targets [8, 15, 16]. Reference [8] proposed a residual attention network in 2017, which enables the classification accuracy to be improved by focusing more on the target information through residual attention networks. A residual attention network is a convolutional neural network containing an attention mechanism, which is constructed by superimposing an attention mechanism in an end-to-end training approach combined with a forward feedback network architecture.

The residual attention network is composed of several attention modules superimposed on each other, and the attention module is divided into two branches: the main branch and the mask branch. The structure of the attention module is shown in Figure 3.

The mask branch contains both upsampling and downsampling layers, which can be both quickly feed-forward scan to collect global information of the image and top-down feedback to combine the global information with the original image features. Each trunk branch has its corresponding mask branch, which is used to learn the attention information of its corresponding layer features, prevent the trunk branch from updating the wrong weight parameters, and can gradually refine the attention features of complex images by superimposing the network structure. The formula for calculating the residual attention block can be shown in the following equation:

(1) $$\begin{array}{c} H_{i,c}=\left(1+M_{i,c}\left(x\right)\right)*F_{i,c}\left(x\right), \end{array}$$

where *F*_*i*,*c*_(*x*) denotes the result of convolutional neural network output and *M*_*i*,*c*_(*x*) denotes the result of mask branch weight output, which takes values in the range of [0, 1], and the closer it is to 0, the closer the output is to *F*(*x*), which can then represent the network as a residual learning network. *M*_*i*,*c*_(*x*) as a feature selector can enhance useful information and suppress undesirable noisy information from the trunk branch, but the increase of attention mechanism makes more parameters in the network, which may cause overfitting and make the training converge slowly.

## 4. Intersection Based on ResNet Network (A-ResNet)

In order to improve the training convergence speed and classification accuracy, the traditional ResNet network model is improved and the A-ResNet network model is proposed and applied to the traffic sign recognition system.

The article "A New Generation of ResNet Model Based on Artificial Intelligence and Few Data Driven and Its Construction in Image Recognition Model" was retracted in 2023. Reasons: unreliable results or conclusions; concerns about the data; concerns about the results or conclusions; concerns about the peer review.

The A-ResNet network is composed of convolutional layer, pooling layer, residual unit, residual attention unit, and softmax layer. Its structural composition is shown in Table 3.

The input image of A-ResNet network has fixed size 224 × 224, and the 112 × 112 feature map is generated after the first convolutional layer and then input to 4 residual units and 3 attention units after the pooling layer is reduced in dimension. Compared with the original ResNet network, we add attention units, adjust the structure of each unit, and add dropout layer, which can speed up the convergence of the loss value of the network training and improve the classification accuracy of the network in recognizing traffic signs.

### 4.1. Improvement of Residual Module in A-ResNet

The structure of the residual unit in the conventional ResNet network is shown in Figure 4(a). The training speed of the ResNet network composed of this structure is slow, and the recognition accuracy is not high, so the structure of the residual unit after adjusting the network to improve the classification accuracy and training convergence speed is shown in Figure 4(b).

The scale normalization layer (BN layer) and the activation layer (ReLU layer) are adjusted to the convolutional layer before the BN layer to normalize the data for stabilizing the network convergence, and then the processed data are input to the Re⁃LU activation function for activation, which can not only increase the nonlinear relationship between the layers, but also enhance the network sparsity and prevent the overfitting phenomenon, and the activated data are input to the convolutional layer. The data after activation is input to the convolutional layer, and the dropout layer is added between the convolutional layers to avoid overfitting of the network parameters.

### 4.2. Improvement of Residual Attention Module in A-ResNet

To address the problem of slow convergence of the residual attention network in the network training phase, an improved residual attention network is proposed in this paper to speed up the convergence of the network training while stabilizing the recognition accuracy. The attention network used is shown in Figure 5.

The basic structures of the residual block, upsampling, downsampling, and jumping branch modules are all consistent with the improved residual unit of this paper. However, the shortcut connection mechanism is not used directly. If the shortcut mechanism is used directly as the structure of the mask branch, it will cause the problem that the gradient of the deep network is not inverted, so the structure of the mask branch is combined with the upsampling and downsampling process, which can obtain the global feature information in the image and convert the extracted global information into a dimensionally consistent feature map. Finally, dimensionally consistent feature maps obtained from the trunk branch and the mask branch are combined by the dot product to form the final output feature map. In the downsampling stage [27], the extracted feature maps are downsampled to a minimum size of 7 × 7 using the maximum pooling layer, and then in the upsampling stage, the feature map dimensions are expanded layer by layer using bilinear interpolation, and the feature maps obtained from downsampling are summed with them to obtain the final feature maps. The purpose of doing so is to combine global and local features to further enhance the characterization capability.

The article "A New Generation of ResNet Model Based on Artificial Intelligence and Few Data Driven and Its Construction in Image Recognition Model" was retracted in 2023. Reasons: unreliable results or conclusions; concerns about the data; concerns about the results or conclusions; concerns about the peer review.

## 5. Results and Analysis

### 5.1. Comparison of Optimization Algorithms

In this study, four algorithms such as SGD, RMsprop, Adam, and Adadelta are compared based on the selection of ResNet-18 as the network model. Due to overfitting, the parameters that converge on the training set are not optimally implemented on the test set [28]. Therefore, in this study, the accuracy and training time of the validation set are chosen as the criteria for comparison, and the experimental data are shown in Figure 6, and it can be seen that SGD performs optimally in both aspects, with the highest average accuracy of 90.99% and the shortest training time of 71.37 min. Therefore, SGD is chosen as the optimal algorithm in this experiment.

### 5.2. Comparison of Model Depth

ResNet uses constant mapping to avoid the “degradation” problem of deep networks and thus can reach very deep network layers. Usually, the increase in the number of layers of the network leads to an increase in the performance of ResNet, but there are also problems such as larger computation, slower convergence, and increased training time [29].

#### 5.2.1. Model Convergence Speed

Convergence in this study means that the accuracy of the network model is infinitely close to the optimal accuracy of the model as the epochs tend to infinity (the maximum value of epochs in this study is 19). ResNet networks of different depths have different rates of approaching their optimal accuracy as epochs become larger. Faster convergence means fast and robust fusion, avoiding overfitting or getting stuck in a local optimum. Progressively deeper colors are used to represent the number of ResNet layers at different depths, and the speed of reaching the optimal accuracy is represented by a line of corresponding color from top to bottom [30]. As shown in Figure 7, all four ResNet models with different depths show no convergence jitter and eventually converge, among which ResNet-18 has the fastest convergence speed and is able to show a stable convergence when the epochs reach 7.

The article "A New Generation of ResNet Model Based on Artificial Intelligence and Few Data Driven and Its Construction in Image Recognition Model" was retracted in 2023. Reasons: unreliable results or conclusions; concerns about the data; concerns about the results or conclusions; concerns about the peer review.

#### 5.2.2. Model Size

At present, as the research on network models continues, the model structure shows a deeper and deeper trend, the complexity of computation deepens, and the size of the model and the amount of memory it occupies increase. Although the hardware facilities of computers are being constantly updated and upgraded, they are still unable to accommodate large-scale complex network models at this stage, which can limit their use on smart devices such as cell phones and computers. Therefore, on the basis of ensuring high accuracy, this study is to find the network models of suitable depth that are lightweight and easy to use on end devices. The sizes of ResNet models with different depths are shown in Table 4. ResNet-18 has a model size of 43.7 MB and requires the least space, which is about 52% of ResNet-34 and 26% of ResNet-101, implying that it takes up less memory, has faster computing time, and is more suitable for mobile.

#### 5.2.3. Equilibrium of Model Identification

The improvement of the balance of the model recognition accuracy is more beneficial to the application of the model in practice and can avoid the problem of poor recognition of specific species. As can be seen from Figure 8, using the average deviation of the recognition error rate of the eight tea samples as the measurement index, the smaller the average deviation value, the stronger the recognition balance of the model.

From Figure 8, it can be seen that the ranking of the balance of the training set is ResNet-18>ResNet-101>ResNet-50>ResNet-34, and the ranking of the balance of the validation set is ResNet-34>ResNet-18>ResNet-50>ResNet-101, ResNet-18. The balance of the recognition in both the training and validation sets is better, and the equilibrium of both the training and validation sets is also better.

In this study, the model performance is measured from four perspectives: convergence speed, size, efficiency, and recognition balance, and finally ResNet-18 is chosen as the basis of the model to build a green tea recognition model, which requires the shortest training time for the fastest convergence speed, effectively maintains the accuracy of image recognition on the basis of the smallest memory occupation and the fastest recognition speed, and performs better in recognition balance. The problem of poor recognition of specific categories can be avoided. As the dataset of this study is more realistic, it proves that the model has a strong practical application capability and breaks through the limitation of many previous studies that cannot fully reproduce the actual diversity. Based on this, the model can be improved in terms of accuracy by using uniform background and field photography to obtain more valid information. In the classification recognition of species by convolutional neural network, the average recognition accuracy of maize [9], chrysanthemum [4], and pepper [1] with different total datasets (3,600, 6,300, and 65,000) and average number of samples per class (1,200, 1,260, and 13,000) reached 95.49%, 95.9%, and 99.35%, respectively (all with clean scenery, with little noise). Therefore, the model can also be optimized and improved by expanding the dataset and selecting more representative team pictures. Green tea species in China are far more than the eight species in this study and can be extended to other tea types in the next study to achieve intelligent recognition of more tea types [31–33].

The article "A New Generation of ResNet Model Based on Artificial Intelligence and Few Data Driven and Its Construction in Image Recognition Model" was retracted in 2023. Reasons: unreliable results or conclusions; concerns about the data; concerns about the results or conclusions; concerns about the peer review.

### 5.3. Green Tea Predicted Classification Results

As shown in Table 5, the low precision, recall, and F-value of Lishui fragrant tea, Lu'an Guapian, bamboo leaf green, and Biluochun indicate that they are more easily confused with other teas, and it can be seen from Figure 9 that Anji white tea and bamboo leaf green, Biluochun, and Lishui fragrant tea are easily confused with each other: in the three validation sets with combined statistics, 10 Anji white teas were misconceived as bamboo leaf green, 12 bamboo leaf green teas were misconceived as Anji white tea, 12 Lishui fragrant teas were misconceived as Biluochun, and 18 Biluochun teas were misconceived as Lishui fragrant tea. This may be due to the similarity in the characteristics of the tea, with Anji white tea and bamboo leaf green both having a certain straight shape, and Biluochun and Lishui aroma tea having a similar curly shape.

The above results may also be due to the existence of some interference in the background which makes some of the tea characteristics not well discriminated, and a higher quality and larger quantity of dataset are needed to support the model for further learning. Data is the driving force of deep learning, and quantity, quality, preprocessing rationality, and labeling accuracy are all important factors. You can expand the dataset by random cropping, random inversion, random brightness transformation, a clean set to take different angles of field shooting to obtain a higher quality dataset. You can also preprocess cropped into smaller and more focused images, and multiple people check the labels to improve labeling accuracy.

## 6. Conclusions

In this study, a new model based on ResNet convolutional neural network to recognize different kinds of green tea was constructed by comparing four different optimization algorithms and investigating the effect of the depth of ResNet model from different aspects. The four optimization algorithms, SGD, RMsprop, Adam, and Adadelta, were compared, and it was found that the stochastic gradient descent (SGD) algorithm required the shortest time and had the highest recognition accuracy.

The article "A New Generation of ResNet Model Based on Artificial Intelligence and Few Data Driven and Its Construction in Image Recognition Model" was retracted in 2023. Reasons: unreliable results or conclusions; concerns about the data; concerns about the results or conclusions; concerns about the peer review.

ResNet-18, ResNet-34, ResNet-50, and ResNet-101 were used to investigate the effect of depth of the ResNet model. ResNet-18 lost only 0.15% accuracy (ResNet-50 had the highest average recognition accuracy of 91.14% and ResNet-18 90.99%). In this study, the heat map of confusion matrix and the respective accuracy, recall, and *F*-value of eight tea types were clarified, and it was found that Lishui fragrant tea, Lu'an Guapian, Zhuyeqing, and Biluochun were more easily confused with other tea types, while Anji white tea and Zhuyeqing, Biluochun, and Lishui fragrant tea were easily confused with each other.

The model constructed in this study is a preliminary application of deep learning in the field of tea variety recognition, and through the selection of optimization algorithm and the exploration of model depth, a better recognition effect is achieved overall. It not only provides a simple and efficient new method for the recognition of green tea species, but also lays a corresponding foundation for further application of deep learning in the field of tea.

## Figures and Tables

**Figure 1:** Partial display of the dataset.

**Figure 2:** Shortcut connection method.

**Figure 3:** Structure of attention module.

**Figure 4:** Residual module before and after improvement. (a) Original residual module. (b) Adjusted residual module.

**Figure 5:** Structure of attention module.

**Figure 6:** Comparison of different optimization algorithms.

**Figure 7:** Convergence speed of ResNet models with different depths.

**Figure 8:** Mean deviation of recognition error rate of 8 green tea species.

**Figure 9:** Heat map of confusion matrix for ResNet-18.

**Table 1:** Number of pictures of different kinds of green tea.

Name	Number	Size range of each image	The size of dataset	The source of images/piece		
				Shopping platform	Social platform	Portal site
Lishui Xiangcha	210	102–1201	61	117	66	27
Xinyang Maojian	204	100–15751	108	152	47	5
Lu'an Guapian	200	102–9088	110	136	53	11
Taiping Houkui	226	114–17780	256	118	108	0
Anji Baicha	224	100–6226	151	134	88	2
Biluochun	210	101–4409	83	180	28	2
Zhuyeqing	199	100–9646	135	101	72	26
Longjing	240	104–11484	298	37	200	9

**Table 2:** Partial presentation of the dataset.

Operating system	Windows10 professional edition
Test platform	Keras
Hardware environment	Intel(R)Core(TM)i7-7700hq CPU@2.80 GHZ 2.80 GHZ
Basic configuration	Anaconda Python3. Version 7

The article "A New Generation of ResNet Model Based on Artificial Intelligence and Few Data Driven and Its Construction in Image Recognition Model" was retracted in 2023. Reasons: unreliable results or conclusions; concerns about the data; concerns about the results or conclusions; concerns about the peer review.

**Table 3:** A-ResNet network model structure.

Arrangement	Output size	A-ResNet
Input layer	224 × 224	
Convolution layer 1	112 × 112	7 × 7, 64
Maximum pooling	56 × 56	3 × 3
Residual element	56 × 56	$\left(\begin{array}{cc} 3\times 3, & 64\\ 3\times 3 & 64 \end{array}\right)\times 1$
Attention unit	56 × 56	Attention ×1
Residual element	28 × 28	$\left(\begin{array}{cc} 3\times 3, & 64\\ 3\times 3 & 64 \end{array}\right)\times 1$
Attention unit	28 × 28	Attention × 1
Residual element	14 × 14	$\left(\begin{array}{cc} 3\times 3, & 64\\ 3\times 3 & 64 \end{array}\right)\times 1$
Attention unit	14 × 14	Attention × 1
Residual element	7 × 7	$\left(\begin{array}{cc} 3\times 3, & 64\\ 3\times 3 & 64 \end{array}\right)\times 2$
Average pooling	1 × 1	7 × 7
Softmax	43 × 1	

**Table 4:** Efficiency and size of ResNet models with different depths.

Model	Identification time per graph	Accuracy %	Size/MB
ResNet-18	0.097 ± 0.0011	90.99 ± 0.37	42.1
ResNet-34	0.112 ± 0.0013	90.94 ± 0.95	82.2
ResNet-50	0.134 ± 0.0009	91.47 ± 0.57	90.2
ResNet-101	0.147 ± 0.001	90.05 ± 0.37	154.5

**Table 5:** Precision, recall, and F-value of the eight green teas.

Classification performance metrics	Precision	Recall	F-value
Lishui Xiangcha	0.85 ± 0.15	0.93 ± 0.008	0.89 ± 0.01
Xinyang Maojian	0.94 ± 0.02	0.95 ± 0.01	0.94 ± 0.01
Lu'an Guapian	0.88 ± 0.01	0.82 ± 0.02	0.85 ± 0.03
Taiping Houkui	0.94 ± 0.03	0.087 ± 0.03	0.91 ± 0.02
Anji Baicha	0.90 ± 0.01	0.88 ± 0.02	0.89 ± 0.04
Biluochun	0.95 ± 0.05	0.97 ± 0.01	0.95 ± 0.02
Zhuyeqing	0.87 ± 0.14	0.95 ± 0.12	0.90 ± 0.12
Longjing	0.98 ± 0.01	0.87 ± 0.02	0.95 ± 0.01

## Data Availability

The dataset used in this paper are available from the corresponding author upon request.
